The article "Efficacy of Cold Atmospheric Plasma Therapy on Chronic Wounds: An Updated Systematic Review and Meta-Analysis of RCTs" was retracted in 2023. Reasons: signs of a paper mill; compromised peer review; unreliable results or conclusions.

# Efficacy of Cold Atmospheric Plasma Therapy on Chronic Wounds: An Updated Systematic Review and Meta-Analysis of RCTs

**DOI:** 10.1155/2022/5798857

**Published:** 2022-10-10

**Authors:** Julan Guo, Yuxing Huang, Bojun Xu, Jiao Yang

**Affiliations:** Hospital of Chengdu University of Traditional Chinese Medicine, Chengdu, China

## Abstract

**Objective:**

A previous meta-analysis has revealed that cold atmospheric plasma (CAP) might not be clinically beneficial to chronic wounds. However, several new randomized controlled trials (RCTs) reported that CAP was an effective treatment option for accelerating wound healing in chronic wounds. The purpose of this review is to incorporate these new results and evaluate the efficacy of CAP in chronic wounds.

**Methods:**

The major databases, including PubMed, Embase, Cochrane Library, and Web of Science, were searched for articles related to CAP treatment in chronic wounds until March 21, 2022. The literature retrieval and evaluation were carried out by two independent researchers.

**Result:**

A total of 13 randomized clinical trials published between 2010 and 2022 were finally included. CAP therapy showed to be more effective in reducing the area of wounds (mean difference (MD): -1.74, 95%; confidence interval (CI): [-3.14, -0.33], *p* = 0.02), compared with non-CAP treatments. The immediate reduction of the bacterial load was higher in the CAP group than in the control group. (MD: -0.37, 95%; CI: [-0.7, -0.05], *p* = 0.02).

**Conclusion:**

No significant changes were found in long-term antibacterial efficacy and pain perception between the two groups. However, more RCTs of excellent methodological quality are required to confirm technical details of the source of AP and the appropriate duration of the treatment with plasma.

## 1. Introduction

Chronic wound is a serious global health issue that results in significant economic and social burdens [1, 2]. Chronic wounds are generally classified into five common types: diabetic foot ulcers, arterial ulcers, venous ulcers, pressure ulcers, and traumatic ulcers. The standard treatment for chronic wounds includes the underlying diseases management, pharmacotherapies, vascular surgery if indicated, and application of absorbent wound dressings on the ulcer lesion. Despite the aggressive therapy described above, the cure rate of chronic wounds is still unsatisfactory, and the recurrence rate is high [1]. Currently, some advanced therapies, including high-intensity laser therapy [3], platelet-rich plasma [4], and stem cell-based therapies [5] are now being tested in clinical studies to see if they might enhance wound healing.

Cold atmospheric plasma (CAP) has been demonstrated to be a potential therapy for wound healing. It refers to a physical plasma (primarily ionized gas) generated at normal atmospheric pressure and ambient temperature, which contains multiple synergistically-acting components such as charged particles, electric currents, ultraviolet radiation, and reactive gas species [6]. The use of CAP in medicine has sparked significant controversy around the world. At present, some studies have been carried out, such as CAP research on cancer [7], antibacterial effect [8], and biological safety [9]. A previously published meta-analysis [10] indicates that CAP fails to bring clinical benefits to chronic wounds healing. However, after that, several new randomized controlled trials (RCTs) have compared the healing effects of CAP on chronic wounds compared to the treatment without CAP. The results indicated that CAP can be an effective treatment option for accelerating wound healing in chronic wounds. The purpose of this review is to incorporate these new results and evaluate the efficacy of CAP in chronic wounds.

## 2. Methods

### 2.1. Inclusion Criteria

The inclusion criteria were set based on the PICO principle:

- *Types of Participants (P)*. Patients with chronic wounds
- *Types of Intervention (I)*. Cold atmospheric plasma
- *Types of control (C)*. Conventional treatments for chronic wounds or placebo
- *Outcomes measures (O)*. (a) Primary outcomes: (i) the reduction of the wound area; (ii) the reduction of the bacterial load; (b) the secondary outcomes: assessment of pain (visual analogue scale) and level of inflammatory cytokines.

Non-RCTs, observational studies, animal studies, case reports, literature reviews, and conference summaries were excluded.

### 2.2. Search Strategy

The literature search was conducted by two reviewers independently. PubMed, Embase, Cochrane Library, and Web of Science databases for all related studies were published before March 21, 2022. The following search strategy was used for the PubMed database: “Wounds and Injuries [MeSH Terms]” or “wound^∗^” or “ulcer^∗^” or “injury” or “injuries” or “Trauma^∗^” AND “Plasma Gases [MeSH Terms]” or “atmospheric pressure glow discharge” or “atmospheric pressure plasma” or “Cold atmospheric plasma” or “Cold atmospheric pressure plasma” or “cold plasma” or “low-temperature plasma” or “non-thermal atmospheric pressure plasma” or “non-thermal dielectric barrier discharge” or “non-thermal gas plasma” or “plasma device” or “tissue tolerable plasma”. Titles and abstracts of retrieved articles were browsed, and irrelevant studies were removed. Full text of potentially eligible studies was obtained and read to identify studies to be included.

### 2.3. Quality Assessment

Two reviewers (GL J and YX H) independently performed the quality assessment of included studies using the Cochrane Risk of Bias Assessment Tool [11], which contained the following domains: randomization sequence generation, allocation concealment, blinding of patients and personnel, blinding of outcome assessments, incomplete data, and selective reporting. Disagreement between the two reviewers was settled via discussion and/or consultation with a third author. Review Manager (RevMan version 5.4) was applied for the risk of bias assessment.

### 2.4. Data Extraction

Data extracted was processed by two reviewers (GL J and YX H), independently using a predesigned standardized form, which contained: name of the authors, region, sample size, age, type of wound, a description of the intervention, control groups, and outcomes. Disagreements were settled through consulting the third reviewer.

### 2.5. Statistical Analysis

All statistical analysis was performed using Review Manager (Ver 5.4). Risk difference (RD) and relative risk (RR) were used as pooled statistic for dichotomous data, and mean difference (MD) was used for continuous data. The 95% confidence intervals (95% CI) of each effect were provided. Heterogeneity among the included studies was assessed using *I*^2^ statistics. An *I*^2^ equal or greater than 50% indicated significant heterogeneity and random-effect model would be applied, otherwise (an *I*^2^ less than 50%), fixed-effect model would be applied. Sensitivity analysis was conducted to assess the robustness of the results via excluding studies of high risk of bias. Funnel plot and Egger's regression test would be applied to assess the publication bias if more than 10 studies were included. A *p* value less than 0.05 would be considered statistically significant.

## 3. Results

### 3.1. Study Selection

Our search strategy retrieved a total of 1,619 articles, and 353 duplicated references were excluded. A total of 1266 studies were initially identified by reading the titles and abstracts. The reasons for the exclusion of the articles are shown in Figure 1. After a comprehensive review of full texts, 71 articles were excluded for the following reasons: conference abstract (*n* = 19), not satisfying inclusion criteria (*n* = 39), and nonrandomized controlled trial (*n* = 15). Finally, 8 papers were included in quantitative synthesis and 5 studies in qualitative analysis. The flow diagram of the study selection process is shown in Figure 1.

### 3.2. General Characteristics of the Included Studies

Characteristics of included studies are presented in Table 1. Eight studies [12–20] were conducted in Germany, three in Iran [21–23], one in Austria [24], and one in Thailand [20]. The 13 included studies involved a total of 477 participants, who were randomized either into CAP treatment group or control group. Patients in the CAP group received both CAP treatment and standard treatment in all of the studies reviewed, although CAP treatment differed significantly in each study. The most-frequently applied standard treatments included debridement, offloading treatment, and wound dressing. There was considerable variation in the type of wound, the source of CAP, and technical details of the parameters applied among the included studies.

### 3.3. Quality of the Included Studies

Quality assessments of included studies are shown in Figure 2. Six studies [12, 17, 20–22] reported the generation of random sequences, and three studies [12, 14, 24] reported allocation concealment. Appropriate blinding of patients was reported in only four studies [12, 14, 17, 19]. Participants in six studies [12, 14, 20–23] were unaware of the group they were assigned, and outcome assessors in four studies [12, 14, 17, 21, 22] were blind to the allocation. Since wound size measurement and bacterial load assessment would be unlikely affected by lack of blinding, the risk of performance and detection bias was considered low. Additionally, because patients who were lost to follow-up and withdrawals were reported in detail, incomplete outcome data were considered to be of low risk of bias. All included RCTs failed to neither prereport the study protocol nor register on any clinical trial registry. This led to unclear reporting bias.

### 3.4. Primary Outcomes

#### 3.4.1. Reduction of Wound Area

Four trials [19, 22–24] reported the reduction of wound area (unit: cm^2^), with 98 patients in CAP group and 91 in control group. As the heterogeneity was detected (*I*^2^ = 18%), a fixed-effects model was used. Meta-analysis showed that CAP treatment was more effective in reducing the wound area [MD = −1.74, 95% CI (-3.14, -0.33), *p* = 0.02, Figure 3], compared with the control group. Sensitivity analysis showed that the removal of any single study did not reverse the results, indicating satisfactory reliability of the outcomes.

#### 3.4.2. Reduction of the Bacterial Load

Three studies [15, 16, 21] reported the immediate reduction of the bacterial load (log *N*^*f*^_*c*_/*N*^*i*^_*c*__,_ where *N*^*f*^_*c*_/*N*^*i*^_*c*_ is the number of colonies after (before) each treatment); 84 patients randomly assigned to the CAP group and 84 to the control group. As the heterogeneity was detected (*I*^2^ = 45%), a fixed-effects model was used. It was shown that the

immediate reduction in CAP group was higher than that in the control group. (MD: -0.37, 95% CI: [-0.7,-0.05], *p* = 0.02, Figure 4(a)). There were two studies [21, 22] reporting the long-term reduction of the bacterial load (log *N*^*f*^_*c*_/*N*^*i*^_*c*__,_ where *N*^*f*^_*c*_/*N*^*i*^_*c*_ is the number of colonies after (before) the entire treatment duration). Significant heterogeneity was considered (*I*^2^ = 52%) so that random-effect model was applied. Meta-analysis showed no statistically significant difference in the long-term antibacterial efficacy between the two groups (MD: 1.86, 95% CI: [-5.36, 9.08], *p* = 0.61, Figure 4(b)). The results of sensitivity analysis test were relatively stable in terms of bacterial load reduction.

#### 3.4.3. Assessment of Pain

Two studies [17, 19] assessed wound pain of patients before and at the end of treatment using the visual analogue scale (VAS), which could score the pain for 0 (no fell of pain) to 10 (most severe pain). As the heterogeneity was statistically significant (*I*^2^ = 78%), a random-effect model was used. The pooled results showed no statistically significant difference between the two groups. (MD: 1.83, 95% CI: [-0.81,4.47], *p* = 0.17, Figure 5).

## 4. Discussion

A previous meta-analysis [10] concluded that CAP treatment did not significantly improve wound healing. However, recently, multiple RCTs have shown that CAP can promote the wound healing. The pooled results revealed that CAP was more effective in accelerating wound healing in chronic wounds compared to the control group. Two main study outcomes were focused in our study: the ability of CAP reducing the area of wounds and the bacterial load in wounds.

Results of quantitative synthesis demonstrated that CAP could be an efficient method to reduce the immediate bacterial load in the wound. Previous studies [25] reported that CAP could generate reactive nitrogen species (RNS) and reactive oxygen species (ROS), which directly affected microorganisms and might cause their inactivation. Reactive nitrogen substances can accumulate on the surface of microorganisms and easily diffuse through cell membranes, resulting in a decrease in intracellular pH. Intracellular pH is important for cell function due to its influences in enzyme activity, reaction rate, protein stability, and nucleic acid structure. Xu et al. [26] reported that helium CAP could reduce staphylococcal biofilm by more than 5 orders of magnitude in only 5 minutes of treatment, indicating that CAP had a short-term antiseptic effect, which was consistent with the results of our results.

A study by Brehmer et al. [18] found a significant bacterial load reduction in chronic venous ulcers in leg following the application of CAP, while no evident reduction was observed in ulcer bacterial strain numbers after an 8-week plasma treatment. Likewise, the results of our quantitative analysis revealed that the antibacterial effects did not seem to last long. Stratmann et al. [12] found that at the end of the entire treatment, the microbial load was reduced in both CAP and placebo treatment groups without significant difference, suggesting that CAP had no long-term antibacterial efficacy.

Another major outcome of this review was the reduction of the wound area. The pooled results showed that in patients with chronic wounds, CAP was more effective in reducing wound area compared to the control group. In another randomized clinical trial [12], CAP therapy showed beneficial effects on the healing of chronic wound as demonstrated by the reduction of wound area and time to wound closure. Moreover, in an RCT [20] that recruited 50 patients with pressure ulcers, the reduction of wound area and decrease in bacterial load were scored and assessed. The wound healing in CAP treatment group showed to be more favorable, compared with control group. First of all, the efficacy of CAP in the reduction of chronic wound areas was attributed to the reduction of bacteria on the wound surface. Bacteria are the most prevalent cause of chronic inflammation that attenuates wound healing. Reactive species produced by CAP are expected to enhance wound healing by reducing bacteria on the surface of the wound [15, 16]. Amini et al. [21] also demonstrated that CAP changed the persistence levels of inflammatory cytokines and growth factors (including IL-1, IL-8, TGF-*β*, TNF-*α*, and INF-*γ*) so that the proliferative phase of the wound was initiated faster which accelerated the healing process. Furthermore, CAP generates some biologically active reactive species, including reactive oxygen species (ROS), which can enhance the synthesis of proangiogenic factors, subsequently promoting wound healing [27]. Hiller et al. [14] reported that expression of several growth factors, such as VEGF-A, FGF-2, and interleukins, might play a crucial role in CAP-mediated granulation promotion, angiogenesis, and reepithelialisation in diabetic foot. These findings might explain why chronic wounds treated with CAP showed a decrease in the area of the wound. In addition, pain intensity was assessed using a visual analogue scale ([VAS]; scale 0-10; 0, no pain; 10, maximum pain) before and after the entire course of CAP treatment. According to meta-analysis, CAP is not more beneficial in terms of relieving pain in patients.

The studies we included concluded that there was no notable adverse effect in either the CAP treatment or control groups. In 2018, Peters et al. [28] pointed out the safety of a new type of CAP device which could be simply applied at home in the future. Besides, there was no adverse effect related to CAP or the procedures, which was consistent with the findings from the studies we included.

Although current systematic reviews indicated that CAP had a positive effect on the treatment of chronic wounds, several limitations should be considered. Firstly, the number of the randomized controlled trials that matched the inclusion criteria was quite small. Secondly, different AP sources and application modes were used in these studies; however, the efficacy of CAP was determined by these parameters. Although the included studies were similar, the type of the patient's wound was not. Thirdly, we did not assess publication bias, considering less than 10 studies for quantitative analysis. In the future, more high-quality RCTs are necessary to evaluate the efficacy of CAP on chronic wounds.

## 5. Conclusion

CAP is an effective treatment for chronic wounds for its effects on reducing bacterial load and wound area, and it will be a promising treatment for chronic wounds. Future research should include the technical details of the source and application parameters of CAP, the appropriate duration of plasma treatment, and the wound characteristics that determine the best treatment.

## Figures and Tables

**Figure 1:** The selection process for the included studies.

**Figure 2:** Risk of bias quality summary [color figure can be viewed at https://wileyonlinelibrary.com/].

**Figure 3:** Reduction of wound area.

**Figure 4:** (a) Immediate reduction of the bacterial load; (b) long-term reduction of the bacterial load.

**Figure 5:** Assessment of pain (VAS).

**(a):** 

Author1 year	Design	Country	Sample size (E/C)	Age (range or mean ± SD)	Type of wound	Intervention group	CAP technical parameters	Control group	Outcomes	Treatment endpoints or treatment duration
Quantitative analysis										
Isbary^15^ 2010	RCT	Germany	38/38	40–94y	VU, AU, DFU, TU	5 min of CAP every day and ST	Microwave 2.46 GHz,86 W; Ar2.2 slm; distance to torch 2 cm	ST	②	Negative bacterial swabs or the wound was healed, or the patient decided to stop.
Isbary^16^ 2012	RCT	Germany	*α*: 14/14 *β*: 10/10	40–85y	AU, VU, TU	2 min of CAP every day and ST	Microwave 2.46 GHz; voltage 50–100 V; power 86 W; Ar2.2 slm	ST	②	Negative bacterial swabs or the wound was healed, or the patient decided to stop.
Heinlin^17^ 2013	RCT	Germany	34/34	64.8 ± 13.4*y*	Skin graft donor site healing	2 min of CAP every day and ST	Microwave 2.45 GHz, 86 W; Ar2.2 slm; distance to torch 2 cm	Placebo and ST	④	Complete healing of the donor site or the patient decided to stop.
Mirpour^22^ 2020	RCT	Tehran	22/22	E: 60.2 ± 5.5*y* C: 54.6 ± 8.8*y*	DFU	CAP (3 times a week for 3 weeks) and ST	Helium gas; voltage 10 kV; frequency 6 kHz	ST	① ③	3 weeks
Moelleken^19^ 2020	RCT	Germany	E1: 14 E2: 13 C: 10	E1: avg65.2y E2: avg66.8y C: avg73.7y	VU, DFU, pyoderma gangrenosum	E1: CAP (1 time a week for 12 weeks) and ST E2: CAP (3 times a week for 12 weeks) and ST	Ar	Placebo and ST	① ④	12 weeks
Amini^21^ 2020	RCT	Tehran	22/22	18–80y	DFU	CAP(3 times a week for 3 weeks)and ST	Helium gas; voltage 10 kV; Frequency 6 kHz	ST	②⑤	3weeks
Samsavar^23^ 2021	RCT	Tehran	10/10	E: 62 ± 6.06*y* C: 59.9 ± 6.23*y*	DFU	CAP (2 times a week for 6 weeks) and ST	Helium gas; voltage 4.5 Kv; frequency 22 kHz	ST	①	6weeks

**(b):** 

Author1 year	Design	Country	Sample size (E/C)	Age (range or mean ± SD)	Type of wound	Intervention group	CAP technical parameters	Control group	Outcomes	Treatment duration
Strohal^24^ 2022	RCT	Austria	39/39	E: 42.58–93.91y C: 42.58–93.91y	VLU, DFU	3 times in the 1st week, twice in the 2nd week, and once per week in the following observation period	CAP-jet treatment (kINPen® med, neoplas med GmbH, Greifswald/Germany)	Best practice wound dressings	①	6 weeks
Quantitative analysis										
Brehmer^18^ 2014	RCT	Germany	7/7	E: 51–85y C: 51–83y	VLU	CAP (3 times per week for 8 weeks) and ST	Frequency 50 Hz, maximum power consumption: 8 VA	ST	① ④	8 weeks
Chuangsuwanich^20^ 2016	RCT	Thailand	23/19	E: 70.75 ± 17.5*y* C: 70.7 ± 1*y*	PU	CAP (once per week for 8 weeks) and ST	Ar; frequency 15–20 Hz; peak voltage was around 6 to 7 kV	ST	Wound and bacterial load reduction is assessed by scores	8 weeks
Stratman^12^ 2020	RCT	Germany	33/32	E: 68.3 ± 9.5*y* C: 68.7 ± 8.8*y*	DFU	CAP (8 times within 2 weeks) and ST	Ar	ST	Wound and bacterial load reduction is assessed by scores	2 weeks
Van Welzen^13^ 2021	RCT	Germany	10/10	74.4 ± 8.1*y*	Skin graft donor site healing	CAP (3 times for 1 week) and ST	CAP was applied using a single dose of 100–240 V and 1.3–8 VA	ST	④	1 week
Hiller^14^ 2022	RCT	Germany	14/13	E: 66.2 ± 11.2*y* C: 68.0 ± 8.6*y*	DFU	CAP (8 times within 2 weeks) and ST	Ar	Placebo and ST	Inflammatory cytokines	

Abbreviations: CAP: cold atmospheric plasma; RCT: randomized clinical trials; E-CAP group; C: control group; y-years; ST: standard treatment; Ar: argon gas; DFU: diabetic foot ulcer; VLU: venous leg ulcer; VU: venous ulcer; AU: arterial ulcer; PU: pressure ulcer; TU: traumatic ulcer. Outcomes: (a) reduction of wound area (cm2); (b) immediate reduction of the bacterial load (log Nfc/Nic, where Nfc/Nic is the number of colonies after (before) each treatment; (c) long-term reduction of the bacterial load (log Nfc/Nic, where Nfc/Nic is the number of colonies after (before) the entire treatment duration); (d) assessment of pain (visual analogue scale (VAS) from 0 (no pain) to 10 (most severe pain)); (e) the level of inflammatory cytokine.

## Data Availability

The data that support the findings of this study are available from the corresponding author upon reasonable request.

## Abbreviations

CAP: Cold atmospheric plasma
RCTs: Randomized controlled trials
MD: Mean difference
CI: Confidence interval
RDs: Risk differences
RRs: Relative risks
ROS: Reactive oxygen species
VAS: Visual analogue scale.
